# Target Characteristics and Voltage Mapping of the Matrix in Idiopathic Premature Ventricular Contractions Originating from the Right Ventricular Outflow Tract

**DOI:** 10.1155/2021/5551325

**Published:** 2021-04-27

**Authors:** Zhiyong Zhang, Xiaofeng Hou, Zhiyong Qian, Jianghong Guo, Jiangang Zou

**Affiliations:** ^1^Department of Cardiology, The First Affiliated Hospital of Nanjing Medical University, Nanjing, Jiangsu 210029, China; ^2^Department of Cardiology, Suqian First People's Hospital, Suqian, Jiangsu 223800, China; ^3^Department of Cardiology, Rugao First People's Hospital, Rugao, Jiangsu 226500, China

## Abstract

**Background:**

The study was aimed at exploring the electrophysiological characteristics (EPS) of the optimal ablation site and its relationship with electroanatomic voltage mapping (EVM) in idiopathic premature ventricular contractions (PVCs) originating from the right ventricular outflow tract (RVOT).

**Methods:**

A total of 28 patients with idiopathic RVOT PVCs underwent successful ablation and EVM using a 3D electroanatomical mapping (CARTO) system.

**Results:**

Both bipolar and unipolar EVM showed a similar band-like lower-voltage area (LVA) under the pulmonary valve in all the patients; 21.4% of the targets were located in the band-like LVA. 42.9% of the targets were at the border of the band-like LVA on the bipolar voltage map, but unipolar mapping showed that 53.6% of the targets were located in the band-like LVA, and 35.7% of the targets at the border of the band-like LVA. A significant difference was found in both unipolar and bipolar voltage values between the regions within 0-5 mm above the optimal ablation site and the other regions. A similar difference was observed only in unipolar voltage values below the optimal ablation site. At the ablation site, there were frequent occurrences of a fragmented wave and voltage reversion in the bipolar electrograms, frustrated falling limbs, W bottom, and a QS configuration width > 150 ms in the unipolar electrograms.

**Conclusions:**

EVM showed that the band-like LVA was an interesting area for the search of the optimal ablation sites of idiopathic RVOT-PVCs, especially the border area. There was focal microscarring around the ablation targets; some characteristics of EPS proved significant for successful ablation.

## 1. Introduction

Premature ventricular contractions (PVCs) without structural heart disease usually originate from the right ventricular outflow tract (RVOT) [1]. Radiofrequency catheter ablation (RFCA) is a safe and reliable treatment for these arrhythmias [2]. However, for some patients who exhibit variable preferential myocardial conduction around the ventricular outflow tract septum or develop dilated cardiomyopathy or arrhythmogenic right ventricular cardiomyopathy (ARVC), RFCA has proven clinically challenging [3].

The pathogenesis of idiopathic RVOT PVCs is currently unclear and is further complicated by the presence of microscars or during the early stages of ARVC [4]. Electroanatomic voltage mapping (EVM) can identify and characterize low-voltage regions and conduction. EVM has been more frequently used for substrate-based mapping and catheter ablation of scar-related ventricular tachycardia (VT) [5]. Studies have revealed that unipolar EVM provides a larger antenna than bipolar EVM to detect fibrofatty substrate involvement of the epi- and midmyocardium, which is commonly present in ARVC patients [6]. The principal objective of this study was to explore the electrophysiological characteristics of the optimal ablation site and its relationship with EVM in idiopathic PVCs originating from the RVOT.

## 2. Materials and Methods

All consecutive patients with idiopathic PVCs with a left bundle branch block pattern and inferior axis with an R/S transition in V3 or later and who were referred for RFCA at Jiangsu Province Hospital and Suqian First People's Hospital were included in the study. PVCs were defined as identically monomorphic and/or couplet PVCs detected by ECG or Holter examination. All included patients signed the informed consent form. The study was approved by the Ethics Committees of the respective hospitals.

All patients underwent detailed cardiac evaluation, including family history, physical examination, 12-lead ECG recording, 24-Holter monitoring, and echocardiography to identify any structural heart disease. Coronary angiography was undertaken to exclude ischemic heart disease, if suspected on the basis of prior investigations. Cardiac magnetic resonance imaging (MRI) was performed to exclude ARVC. Finally, the patients who underwent EVM of the RVOT during sinus and those with successful ablation sites below the pulmonary valve were enrolled in the study.

Electrophysiological study (EPS) and radiofrequency ablation procedures were performed in all patients after written informed consent was obtained. Antiarrhythmic drugs were discontinued in all patients for more than five half-lives before EPS. Some patients presented with or without spontaneous PVCs at preoperative baseline. To determine the eligibility of patients, clinical PVCs were induced by administering routine programmed electrical stimulation or intravenous administration of isoprenaline (1-5 *μ*g/min). For voltage mapping during sinus rhythm and activation mapping during PVC occurrence, a 3D electroanatomical mapping system (CARTO) with a deflectable tip electrode (Navistar Thermocool, Biosense Webster)—either a 4 mm nonperfused diagnostic ablation catheter or a Navistar catheter with a 3.5 mm deflectable tip electrode (Navistar Thermocool, Biosense Webster)—was used.

At least 50 measurements were obtained from the sinus rhythm of the patients to construct a high-density electroanatomical mapping model of the ventricular outflow tract. The pulmonary valve location was estimated by the guidance of biaxial fluoroscopy and right ventriculography. For the cases mapped using the CARTOXP system, the merged images from cardiac computer tomography and electrical mapping were used to confirm the location of the pulmonic valve. The bipolar electrogram signals were filtered at 30-500 Hz, and the unipolar signals at 1-240 Hz were recorded at an ECG rate of 100 m/s. Wilson's central terminal was used as the second electrode for unipolar recordings. Recordings were collected and integrated into the map, where the variability of the cycle length was <2%, local activation time (LAT) was <3 mm, and the maximum beat-to-beat difference in the location of the catheter was <4 mm, respectively. During the ablation procedure, the catheter was moved to coincide with the motion of the beating heart to optimize the consistency of the results.

Normal amplitude electrograms (bipolar ≥ 1.5 mV; unipolar ≥ 6.0 mv) were represented in the electroanatomic CARTO map by a purple color. Red color indicated a dense scar, which was arbitrarily defined as the bipolar signal amplitude < 0.5 mV or unipolar signal amplitude < 3.5 mV, according to the previously reported criteria [5, 6]. The intermediate colors represented the lower-voltage area (LVA) and the borderline between the normal areas and LVA, which was defined as the LVA “border.”

Activation or pace mapping was used to identify the ablation target. The position of the earliest local activation during arrhythmia, or the amplitude of the surface ECG with pace mapping displayed on at least 11 leads, needed to be consistent with the spontaneous arrhythmic ECG. The specifications for ablation using different catheters were as follows: (1) 4 mm catheter, temperature = 50-60°C, and radiofrequency energy = 50 W delivered continuously for 60–120 s and (2) Navistar catheter with a 3.5 mm deflectable tip electrode infused with saline, temperature = 42°C, and radiofrequency energy = 50 W for a duration of 60–120 s. Subsequently, routine programmed electrical stimulation or intravenous isoprenaline was administered. Acute ablation was considered successful if there was no induction of clinical ventricular prematurity or ventricular tachycardia. No recurrence after 30 minutes of observation represented the actual target of arrhythmia. The target region was divided into two anatomical subdivisions according to the electroanatomical morphology: RVOT as the septum (anterior, middle, and posterior) and the free wall (anterior, middle, and posterior). The electrophysiological characteristics determined by unipolar and bipolar electrograms of the target, as well as the voltage values at various distances from the target (5 mm, 5-10 mm, and 10-15 mm), were recorded and analyzed.

All data were statistically analyzed using the SPSS version 16.0. Variables are expressed as mean ± standard deviation (SD). For comparison of samples, a *t*-test was conducted. Attribute data are displayed as a rate. The chi-squared or Fisher exact test was used to compare samples. Results are considered statistically significant if *P* < 0.05.

## 3. Results

A total of 28 patients, aged 40.6 ± 11.9 years (7 males and 21 females) with the following clinical features, were included in this study: ejection fraction (EF): 63.6 ± 3.9%; 24-hour PVC count: 30,687.5 ± 17,234.9; and PVC burden: 25% ± 10%. Successful ablation was acutely achieved in all patients with no arrhythmia recurrence before hospital discharge or in the late 6 months' follow-up phase without the use of antiarrhythmic drugs.

The average distance of the optimal ablation site from the pulmonary valve annulus was 19.2 ± 8.9 mm. 75% (21/28 patients) of the targets were located in the septum, and 52% (11/21 patients) of the targets were in the anterior septum. Among the free wall targets, 85% (6/7 patients) were located in the anterior free wall (Figure 1).

For the bipolar electrogram characteristics of successful ablation sites, 78.5% (22/28) of patients displayed no specificity in their QRS morphology with electrogram morphology. As displayed in Figure 2(a), the distal and proximal polarities were reversed (distal Ab1-2 pointing vertically downward in the initial part of the waveform and Ab3-4 vertically upward) in 11% (3/28) of patients. The fragmented wave pattern was noted in 11% (3/28) of patients (Figure 2(b)). The electrogram of the ablation site proceeded to 29.28 ± 6.55 ms from the onset of the QRS complex during the PVCs.

For the unipolar electrogram characteristics of successful ablation sites, all (28/28) patients presented a QS complex, 57% (16/28) of patients displayed a frustrated descending limb, and 32% (9/28) of patients showed a W shape in the QS electrogram morphology. The width of the unipolar QS complex was 156.8 ± 17.7 ms. Unipolar electrogram characteristics of successful ablation sites are shown in Figures 2(c) and 2(d).

Both unipolar and bipolar maps displayed band-like low-voltage regions below the pulmonary valve during sinus rhythm (Figure 3). For the optimal ablation sites, the unipolar voltage was 9.79 ± 5.20 mV and the bipolar voltage was 2.86 ± 2.05 mV. A significant difference (*P* = 0.001) was observed between the unipolar and bipolar voltage values.

On the bipolar map, 21.4% (6/28) of patients had targets located in the band-like LVA below the pulmonic valve, 42.9% (12/28) of patients had targets located at the border of the band-like LVA, and 35.7% (10/28) of patients had targets below the band-like LVA border (in the normal area). On the unipolar map, 53.6% (15/28) of patients had targets located in the band-like LVA, 35.7% (10/28) of patients had targets at the border of the band-like LVA, 3.6% (1/28) of patients had targets below the band-like LVA border, and 7.1% (2/28) of patients had targets above the band-like LVA (in the scar area) (Figure 3). For the areas above the target, there was a significant difference between 0-5 mm and the others for unipolar voltage values (*P* < 0.05), but there were no significant differences between 5-10 mm and 10-15 mm (*P* > 0.05). Similar findings were observed for bipolar voltage values.

For the areas below the target, there was a significant difference between 0-5 mm and the other areas for unipolar voltage values (*P* < 0.05), but there were no significant differences between 5-10 mm and 10-15 mm (*P* > 0.05). We did not observe a similar relationship in the three areas for the bipolar voltage values (*P* > 0.05). The unipolar and bipolar voltage values of various areas are shown in Figure 4 and Table 1.

## 4. Discussion

The present study explored the electrophysiological characteristics of optimal ablation sites using unipolar and bipolar electrograms. We also investigated the EVM of the matrix around the targets to identify the optimal ablation site for idiopathic PVCs originating from the RVOT, which remains a clinical challenge in some patients.

Our data are consistent with previous clinical findings, as targets in 75% of patients were found in the septum. Additionally, the maximum targets in the septum and free wall were located anteriorly [7]. Our observations are consistent with those of Yu et al. [8].

In the present study, all patients underwent activation mapping. A previous activation mapping study suggested a mean activation time of -23 ms before the onset of the PVC QRS complex as a negative predictive value for ablation on the catheter bipolar electrogram [9], but we report the activation time for optimal ablation site as −29.28 ± 6.55 ms before the onset of the PVC QRS complex. We also found that the phenomenon of reversion of the distal and proximal polarity of the ablation catheter and fragmented wave is not rare, since this occurred in 11% of the patients in this study. Furthermore, Fisher et al. [10] first reported a QS wave on the unipolar electrogram in addition to the frequent observations of a frustrated falling limb with W-shaped QS waves [10]. van Huls van Taxis et al. [11] reported that the reversed polarity has 81% sensitivity in distinguishing a successful ablation target, but the prediction sensitivity reversed polarity is lower than that of unipolar QS (85%) and LAT (85%). However, the specificity of reversed polarity has also been reported as 93% for detecting a successful ablation target, which is far higher than that of LAT (71%) and unipolar QS (35%) [11]. Additionally, the combined use of reversed polarity and LAT offered 86% accuracy for identifying successful ablation targets [11]. A QS configuration is observed only if the ablation catheter is present at or close to the site of ectopic focus, which is beneficial when the information provided by a unipolar electrogram contains far-field signals referring to a large area [11]. The present study also observed a QS configuration in a 10-15 mm radius surrounding a successful ablation site. For excluding far-field signals, ablation under the guidance of rapid negative deflections is helpful [11]. This concept is also consistent with the results of Pang et al. [12]. Moreover, Huang *et al.* [13] demonstrated that the sensitivity and specificity in successfully predicting an ablation target when guided by electrogram with a frustrated descending limb were 72.6% and 91.7%, respectively. This suggests uneven electrical conduction in local activation mapping, small-sized myocardial sleeve tissues, and slow propagation of the depolarizing impulse that leads to limited characteristics on the unipolar electrogram. This study also found a W-shaped bottom unipolar QS complex when a width > 150 ms was displayed on the electrogram of successful ablation sites of several patients. Considering the evidence, the combination of unipolar and bipolar ECG can contribute to efficient identification of target ablation sites in clinical practice.

In the present study, both bipolar and unipolar EVM revealed a band-like LVA below the pulmonary valve in all patients. Both the bipolar and the unipolar map showed that the majority of the optimal ablation sites were located in the band-like LVA, especially at the border of the band-like LVA in the bipolar map. These results are consistent with multiple publications. Huang et al. [14] and Yamashina et al. [7] discovered that the original site of RVOT arrhythmia is more likely to appear in the translational voltage zone and at the edge of the LVA. Wang *et al.* [15] found that 91.7% of patients had successful ablation targets in the transitional voltage zone below the pulmonary valve, while Lin *et al.* [16] reported that the ablation targets in 67% of patients were found in the transitional voltage zone. Furthermore, Liu *et al.* [17] found that the isolated diastolic potentials (IDPs) can be recorded in all patients with ROVT arrhythmia. Together, these studies demonstrate that the translational voltage zone is comprised of normal cardiac muscle and fibrous tissue, including a mixture of healthy and damaged cardiac muscles, resulting in heterogeneous conduction of cardiac pacing.

After comparison of voltage mapping in various regions at different distances from the target, we found that bipolar voltage mapping showed a significant difference between the 0-5 mm radius and other areas only above the target; however, unipolar voltage mapping showed a significant difference between the 0-5 mm radius and other areas both above and below the targets. This demonstrates that the unipolar EVM provides a larger antenna than bipolar EVM to detect fibrofatty substrate involvement in the epi- and midmyocardium. These findings are consistent with the fact that the existence of an inactivated region of heterogeneous conduction around the pacing site results in ROVT-PVCs. Therefore, the endocardial optimal ablation site is located mainly in the breakout site or at the exit of the PVC origin. Finally, the present study demonstrated the presence of focal microscarring around an inner ectopic focus, equivalent to a catheter tip width radius from a different perspective.

All patients were successfully ablated through positioning the ablation catheter below the pulmonary valve. Due to the nonspecific landmarks or scope to determine the location of the pulmonary valve, a combination of X-ray imaging and polarity characteristics can be beneficial. Therefore, we used the threshold of the endocardial bipolar electrogram to identify the pulmonary valve, which is considered the junction between the scar tissue and the low-voltage region at the electroanatomical boundary below the pulmonary valve. The low-voltage region represented the translational zone below the pulmonary valve. Although the anatomical structures are different in the pulmonary sinus, above or below the pulmonary valve, all were in the abnormal voltage zone on 3D voltage maps, which confirmed our findings and conclusions.

A limitation of the present study is the low sample size with traditional mapping methods that underwent ablation. Thus, further studies with new features of mapping methods (such as high-density mapping catheters and contact force catheters) are required to confirm these findings. For inclusion in the study, the participants were evaluated by echocardiography and coronary angiography to exclude high-risk patients with common ischemic and nonischemic heart diseases. However, the cardiac MRI failed to identify patients with a distribution of ablation targets in the low-voltage zone, and we were therefore unable to exclude patients with potential illness, such as ARVC and cardiac nodal disease.

## 5. Conclusions

In summary, the optimal ablation sites of idiopathic RVOT arrhythmias are primarily located in high-risk areas, especially at the border of the band-like LVA on the bipolar voltage map. For focal microscarring around the ablation targets, the ectopic focus is located in the mid- or epimyocardium. The addition of EVM to the intracardiac electrophysiological study proved significant for successful ablation.

## Figures and Tables

**Figure 1:** Successful ablation target locations. 75% (21/28 patients) of the targets were located in the septum, and 52% (11/21 patients) of the targets were in the anterior septum. Among the free wall targets, 85% (6/7 patients) were located in the anterior free wall.

**Figure 2:** Electrogram characteristics of successful ablation sites: (a) duration and morphological characteristics of the premature QRS complex on bipolar ECG at the ablation target; (b) fragmented wave on a bipolar ECG at the ablation target; (c) QRS width and morphological characteristics of a unipolar ECG at an ablation target; (d) QRS morphology on a unipolar ECG showing a W shape at the ablation target.

**Figure 3:** Relationship between the target and band-like lower-voltage area (LVA) in different regions (PA: posteroanterior; RL: right lateral; LL: left lateral). The blue dot denotes the target, which is at the border of the LVA on the bipolar voltage map and in the LVA on the unipolar voltage map.

**Figure 4:** Three different areas above and below the target on the unipolar and bipolar maps.

**Table 1:** Comparison of unipolar and bipolar voltage values in various areas.

Voltage	Areas (above or below the target, mm)	Voltage (mV) (mean ± SD)	*P* value
Unipolar	0-5 mm (above)	4.52 ± 2.41	0.001^#^
	5-10 mm (above)	3.34 ± 1.69	0.001^∗^
	10-15 mm (above)	3.02 ± 2.04	0.999^¥^
	0-5 mm (below)	5.39 ± 2.67	0.001^#^
	5-10 mm (below)	6.38 ± 2.67	0.002^∗^
	10-15 mm (below)	7.25 ± 3.11	0.999^¥^
Bipolar	0-5 mm (above)	1.68 ± 1.78	0.006^#^
	5-10 mm (above)	1.35 ± 1.64	0.006^∗^
	10-15 mm (above)	0.84 ± 1.23	0.999^¥^
	0-5 mm (below)	3.18 ± 1.99	0.999^#^
	5-10 mm (below)	3.42 ± 1.55	0.999^∗^
	10-15 mm (below)	3.91 ± 2.08	0.999^¥^

^#^Comparison of the 0–5 mm radius above the target and 5–10 mm radius above the target or comparison of the 0–5 mm radius below the target and 5–10 mm radius below the target; ^∗^comparison of the 0–5 mm radius above the target and 10–15 mm radius above the target or comparison of the 0–5 mm radius below the target and 10–15 mm radius below the target; ^¥^comparison of the 5–10 mm radius above the target and 10–15 mm radius above the target or comparison of 5–10 mm radius below the target and 10–15 mm below the target.

## Data Availability

All data generated or analyzed during this study are included in this article.
